# Blockchain and Fog Computing in IoT-Driven Healthcare Services for Smart Cities

**DOI:** 10.1155/2022/9957888

**Published:** 2022-01-25

**Authors:** M. M. Kamruzzaman, Bingxin Yan, Md Nazirul Islam Sarker, Omar Alruwaili, Min Wu, Ibrahim Alrashdi

**Affiliations:** ^1^Department of Computer Science, College of Computer and Information Sciences, Jouf University, Sakakah, Saudi Arabia; ^2^School of Public Administration, Sichuan University, Chengdu, China; ^3^School of Political Science and Public Administration, Neijiang Normal University, Neijiang, China; ^4^Department of Computer Engineering and Networks, College of Computer and Information Sciences, Jouf University, Sakakah, Saudi Arabia

## Abstract

Nowadays, technology has been evolving rapidly. Due to the consequent impact of smart technologies, it becomes a ubiquitous part of life. These technologies have led to the emergence of smart cities that are geographic areas driven by advanced information and communication technologies. In the context of smart cities, IoT, blockchain, and fog computing have been found as the significant drivers of smart initiates. In this recognition, the present study is focused on delineating the impact and potential of blockchain, IoT, and fog computing on healthcare services in the context of smart cities. In pursuit of this objective, the study has conducted a systematic review of literature that is most relevant to the topic of the paper. In order to select the most relevant and credible articles, the researcher has used PRISMA and AMSTAR that have culminated in the 10 most relevant articles for the present study. The findings revealed that IoT, blockchain, and fog computing had become drivers of efficiency in the healthcare services in smart cities. Among the three technologies, IoT has been found to be widely incorporated. However, it is found to be lacking in terms of cost efficiency, data privacy, and interoperability of data. In this recognition, blockchain technology and fog computing have been found to be more relevant to the healthcare sector in smart cities. Blockchain has been presented as a promising technology for ensuring the protection of private data, creating a decentralized database, and improving the interoperability of data while fog computing has been presented as the promising technology for low-cost remote monitoring, reducing latency and increasing efficiency.

## 1. Introduction

The world has recently experienced immense urban growth in recent years, which is mainly attributed to the continual increase in the world's population. It is also evident from the fact that 54% of the individuals are living in cities as compared to 46% who are living in the rural areas and it is expected that it will continue to increase to 66% by the year 2050. To address urbanization, the urban planners and concerned authorities focus on emerging technologies for cutting the costs, specifically by ensuring optimal utilization of resources and creating a sustainable environment for living [1]. In this regard, Karale and Ranaware [2] and several other researchers have highlighted that big data, the Internet of Things (IoT), artificial intelligence, machine learning, multimedia, blockchain, cyber-physical system, and cloud computing have gained prominence due to their wide-ranging benefits in different domains [3–8]. It is anticipated that the application of these technologies would contribute to the development of fully automated secure smart cities [9–14].

According to Treiblmaier et al. [15], a “smart city” is the densely populated geographical area that uses emerging information and communication technologies for connecting the physical components, thereby, enhancing the information flow, increasing the overall efficiency of the city operations, and improving quality of life of the citizens. The underlying concept is to create an environment where technology is fully embedded within the city for addressing the issues of urbanization, specifically by adding high-value services. In this regard, Burnes and Towers [16] have highlighted that the essence of smart cities lies in the infrastructural and technological complexities. Therefore, the designers of smart cities seek innovative ways to develop such technological infrastructure that is capable of catering to the social, environmental, and economic needs of people.

Al-Azzam and Alazzam [17] have argued that smart cities have several components, among which smart healthcare has gained immense popularity in the past years, particularly to ensure the provision of quality healthcare services to the citizens. In particular, the concept of smart health (s-health) is related to assuring the provision of health services through the utilization of efficient networks and technological infrastructure of smart cities [18]. It is significant to note that there is a difference between m-health and s-health, as s-health aims to improve m-health by adding sensing abilities in smart cities. The healthcare sector has been experiencing a substantial increment in the volume of medical data of the patients shared between the insurance companies and the healthcare providers, which has resulted in the emergence of data-driven healthcare models [19]. Since healthcare services are producing an enormous amount of information, therefore, strong security mechanisms like access controls are required to preserve the privacy of individuals [20]. This has eventually developed the need of exploiting emerging technologies like blockchain, IoT, and fog computing for ensuring faster and safe access to healthcare data, thereby, enhancing the quality of healthcare services [21].

The current study aims to analyze the impact of blockchain, IoT, and fog computing, specifically in the context of healthcare services in smart cities. This particular topic is highly relevant as urbanization has developed the need to improve healthcare services by integrating smart technologies. It is anticipated that such initiatives would result in the establishment of smart cities, hence, providing the citizens with enhanced quality of healthcare services. However, Dwivedi et al. [21] have highlighted that hackers tend to seek to gain access to health information for identity theft, as medical records are present in different forms like reports, videos, images, and raw data whose integrity is crucial. Since the emergence of bitcoin, the possibilities of utilizing the blockchain have become endless as the underlying technology can serve several benefits. The blockchain has a low cost, while its security is based on a proof of work concept where the transaction is only considered valid when a sufficient amount of computational work has been performed for solving the cryptographic puzzles which are done by the authorizing nodes. The inability to delete or change the information present in the block has eventually regarded blockchain as the best technology which can be exploited for the healthcare system in smart cities [22–24].

To conceptualize, Zheng et al. [25] have defined blockchain as the distributed database of the transaction on a scalable network that the authorized parties can only access on the web. The authorized parties verify the transactions stored in public databases on the network. Moreover, the transaction information that is stored on the blockchain is protected by cryptography and, thus, can never be erased. Hence, it is saved from loss and alteration. All the transaction blocks are linked/chained with each other resulting in a sequence of blocks. It implies that as the number of the transaction blocks increases, the chances of data getting altered decreases [26]. The hashing is applied to the transaction information to convert them into an encrypted form. In case of any change made to the previous block, the hash of the block changes the hash of the subsequent blocks. This is why any change made to any block can easily be spotted and rejected. The process of the chained block is demonstrated in Figure 1.

Figure 2 illustrates the structure of the blocks in the blockchain.

Atzori et al. [27] have defined the Internet of Things (IoT) as the network of devices that interacts with each other through machine to machine (M2M) communications, hence, allowing the collection and exchange of data. The technology combines a range of communication and network devices, sensors, cloud, services, systems, etc. [28]. These technologies leverage their computing power and interconnectedness to exchange vast amounts of data [29]. The IoT architecture is comprised of various layers of technologies and communication devices. There is no standard or universally agreed-on architecture for the IoT system. Different IoT systems can be different from each other based on the range of sensors, communication devices, networks, objects, etc. [30].  Figure 3 illustrates the architecture of the IoT system.

Currently, IoT has transformed the healthcare sector by enabling healthcare professionals to exploit the benefit of remote health monitoring where doctors can monitor noncritical patients at home instead of in a hospital. This feature contributes to reducing the workload on hospital resources. IoT healthcare systems have been recently developed for serving different purposes like diabetes management, rehabilitation, assisted ambient living (AAL) for elderly individuals, etc. [32]. These IoT solutions mainly employ the use of mobile devices (smartphones) along with the gadgets like sensors, Bluetooth for near field communications, smart contact lenses, blood pressure monitors, smartwatches, and other tools. These gadgets are connected to a particular network for sharing the processed information between the patient and healthcare provider [33].

Tariq et al. [34] have stated that the existing infrastructure of the healthcare sector is not sufficient for which blockchain is expected to facilitate data collection from different sources and to store them in the transaction audit log. This audit log can be used to track the transactions for accountability and transparency during an exchange of medical records between the insurance companies and healthcare providers. Moreover, blockchain-based solutions for healthcare can assist patients in identifying and tracking the modifications that have been made in their medical data. Besides this, patients can also control the use of their medical data by permitting certain parties who can only view them instead of storing and modifying the data. This would eventually change the current practices where only healthcare providers are the owners of patients' data, thus, effectively addressing the issues associated with security, trust, privacy, and integrity.

Karale and Ranaware [2] have stated that blockchain technology enables creating a single healthcare record for a particular individual, which can be made available at any time during health emergencies. The underlying idea is to ensure the decentralization of medical records, hence, facilitating the patients to freely visit the health consultant instead of being worried about carrying their health records with them. The faster access to the health data has allowed the healthcare professionals to detect the warning signs of serious illness in the early stages of the diseases, thus, enabling them to save several lives [35]. This aspect has become increasingly important in recent times, where COVID-19 has hit hard the densely populated areas. Recently, Spanish researchers have used blockchain technology to support healthcare officials in controlling COVID-19 spread, specifically by enabling them to make smarter decisions related to a pandemic like social distancing and quarantine measures. Moreover, the capabilities of blockchain have also contributed to streamlining the processes of healthcare, tracking the COVID-19 patients, and reducing the extensive workload of hospitals that were continually increasing due to high transmission of the virus, thus, depicting the relevance of shifting toward smart cities approach [36]. Succinctly, it can be articulated that the present research study would significantly contribute to analyzing the role and importance of implementing blockchain technology in the healthcare system of smart cities.

Ahmed et al. [37] have discussed that IoT technology offers emergency response and recovery support in critical situations. Since unpredictable disasters have the capability of completely affecting and closing down the infrastructure of human society, in these times, IoT solutions provide real-time support [38, 39]. It includes vehicle tracking and coordination between the healthcare workers and rescue workers and patient monitoring. The timely identification of warning signs allows healthcare professionals to arrange ambulatory services with fast routing features to reach the nearest hospital or clinic for emergency healthcare services. Thus, this research study will assess the role and impact of IoT on the healthcare sector of smart cities.

Besides IoT and blockchain, fog computing has also gained substantial popularity in the past few years. Fog computing is an architecture based on handling the data at network edges to address the downsides of cloud computing [40, 41]. Due to these features, fog computing has prominent applications in smart cities. Since the sensing processes are improved in fog computing, data processing is done in a speedy manner that reduces latency [42]. In simpler words, Cha et al. [43] have defined fog computing as a virtual platform through which the computing device can exchange, process, and save data on a cloud computing data center. It is the network connection between the cloud data center and the edge device.  Figure 4 illustrates the structure of fog computing.

Fog computing has gained significant prominence in the time-sensitive healthcare applications that require immediate response like remote patient monitoring applications and, therefore, are employed alongside IoT gadgets [44]. Al-Khafajiy [45] has discussed that fog computing provides the benefits of storage, networking, and computing services between the devices. Thus, the healthcare sector is benefited through a decrease in latency and an increase in consistency as compared to cloud solutions. The application of fog computing, i.e., remote monitoring of healthcare patients—supported by sensors—has replaced the manual supervision procedures of in-hospital follow-ups and has positively impacted the survival of patients. The ability to gain correct information about the patients and process it speedily has enabled healthcare professionals to enhance the quality of medical healthcare services. Besides, fog computing can improve the privacy of the patient's data as it analyzes the sensitive data on the local gateway instead of the data center [46]. Thus, the improved security mechanisms of fog computing have gained prominence in the healthcare sector, for which the present research is intended to study the effect of fog computing on healthcare services in smart cities to expand its broader applications.

The methodologies used in this research are a systematic qualitative review along with the application of AMSTAR and PRISMA tools. AMSTAR is mainly used for identifying the quality of the study through the questions generated by the tool. However, PRISMA is applied for narrowing down the research studies used for the review. The remainder of the paper is described as follows: Section 2 explains the materials and methods; Section 3 deals with results; Section 4 interprets with discussion; Section 5 concludes the paper with future research direction.

## 2. Materials and Methods

### 2.1. Research Approach and Design

The present paper incorporates a qualitative research approach in order to undertake a periodic and qualitative synthesis of the existing literature pertinent to the topic of blockchain, IoT, and fog computing for healthcare services in smart cities. The rationale for the selection of the methodology is embedded in the research philosophy of interpretivism, whereby the researcher would interpret the elements of the research qualitatively rather than relying on quantitative data [47]. In this regard, the study will be based on the scientific review of the seminal work pertinent to the selected topic. The researcher would review, analyze, and evaluate the research process and the findings and the results of the relevant seminal work.

### 2.2. Review of the Seminal Work

In order to synthesize the existing literature, the researcher intends to incorporate a systematic literature review with the incorporation of which the researcher will collate the empirical literature [48]. The researcher would identify the most relevant research papers and conduct a critical analysis of the selected material. In this regard, the paper will be based on the synthesis of a number of credible and relevant journal articles and other studies on relevant topics from reliable and credible secondary data sources such as Google Scholar, EBSCOhost, JSTOR, and Emerald. It implies that the selected material for the systematic review must correspond to the topic “blockchain, IoT, and fog computing for healthcare service in smart cities.” In order to find such articles, relevant keywords will be used, such as IoT, blockchain, and fog computing. Moreover, to ensure that the findings of the present paper are accurate and up to date, it is intended to select articles between the period 2015–2020.

### 2.3. Criteria for the Selection of the Seminal Work

In order to conduct a systematic literature review, it is imperative to develop a selection criterion prior to the identification of the articles selected for the study. In this regard, for the present study, the researcher intends to analyze at least 10 relevant articles extracted from credible sources. The selected articles must be in line with the following criteria:

- The selected articles must be written and published from 2015 to 2020
- The topics of the articles must correspond to the topic “blockchain, IoT, and fog computing for healthcare service in smart cities”
- The article can be based on a qualitative or quantitative study
- Grey literature such as technical reports, conference papers, or websites is not included in the systematic review of this study
- The articles must be sourced from reliable and credible sources
- The articles must be based on the author's original work and must include an abstract, a research process, and a clear conclusion

### 2.4. Quality Assessment and Data Extraction

It is important to be mindful that studies, including systematic reviews pertinent to the healthcare sector, have been increasing with a number of researchers trying to contribute to the literature. However, such systematic assessments are subject to a variety of biases that contain, increasingly, nonrandomized intervention trials. It is critical for consumers to be able to differentiate between high-quality reviews. Many methods have been developed to analyze specific facets of feedback, but there are few systematic tools for critical evaluation [49]. In this regard, in order to assess the quality of the selected articles and to ensure that the articles used for the review are of high quality, the author has incorporated the AMSTAR tool and PRISMA approach. With the incorporation of the AMSTAR tool, the investigation of methodological and the analytical consistency of the research has been conducted. It enabled the author to conduct a quality assessment of the papers pertinent to “blockchain, IoT, and fog computing for healthcare service in smart cities.”

Quality assessment is shown in the appendix. Moreover, with the incorporation of the PRISMA approach, the information pertinent to each of the selected articles is critically evaluated, taking into consideration any bias in the findings and the results of the study [49]. The articles that were shortlisted after using the AMSTAR tool were further analyzed based on the predetermined factors (by PRISMA checklist), including the year of publishing. For the present report, the author collected 30 papers through the initial search. After the filtering process, 10 articles were selected for the current review. It has been ensured that the selected articles are based on the relevant research area and research question, have carefully addressed the research topic, and generate relevant findings. Since the present study is based on a contemporary research area with technology, not much literature could be found. Thus, in order to ensure that only credible and the most relevant studies are selected for the present review, a small number of the articles are selected.  Figure 5 demonstrates the PRISMA process for the present study.

## 3. Results

The incorporation of advanced digital technologies has led to the emergence of smart city initiatives that are geographical regions integrating a wide range of information and communication technologies. The study by Al-Azzam and Alazzam [17] states that the introduction of ICT has contributed to the evolution of smart cities. Similarly, the usage of mobile devices and ICT for health-related problems would lead to the appearance of ubiquitous surveillance of patients and health services using e-health and smart health [50]. With the incorporation of smart health, healthcare institutions can be benefited from various opportunities. For instance, it would help in the identification of the circumstances that need intervention, identification of the patients that are suffering from chronic diseases and need attentive care, and modification of the laws and regulations by taking into consideration the laws enforced in the city or the district as well as the environmental condition of the locality [17].

One of the significant technologies that have been incorporated to make healthcare services smarter is IoT technology. As per the findings of Baker et al. [30], with the incorporation of the IoT, healthcare systems can leverage big data and self-learning systems. Thus, such intelligent systems can be used to ensure smarter management of healthcare practices. For instance, various anomalies can be analyzed, culminating in identifying the specific actions to be taken to provide appropriate healthcare to the patients. Building on the patient's data, the care providers can ensure the provision of personalized care to the patients as well as the standardization of various practices.

Similarly, Perera et al. [42] state that remote healthcare surveillance has been made possible by powering healthcare practices through IoT technology. Care providers can remotely track noncritical patients, mitigating demand on in-house hospital services such as doctors and beds [50, 51]. It may also be used to provide greater access to services for those living in remote areas or to make it easier for disabled people to live comfortably for longer at home. Essentially, access to healthcare services should be increased without reducing the burden on healthcare facilities, and people should now have more control of their health.

However, it is also found that healthcare systems have been incorporating IoT technology to manage large volumes of data [52]. Baker et al. [30] posited that systems powered by IoT technology might present a threat to the protection and the privacy of the patients' personal data. Unauthorized access to such devices can result in theft of the data and breach of data privacy regulations. In this regard, the blockchain has been found to be yet another driving force of smart city initiatives. As per the study by Treiblmaier et al. [15] in the healthcare sector, large volumes of patient data are exchanged between the healthcare institutions and the insurance agencies. This has resulted in the advent of healthcare models powered by data. Hence, healthcare systems require high confidentiality and access control [53, 54]. The study pointed out that blockchain technology paves the way for smart healthcare with which such volumes of data can be smartly handled along with the issues pertinent to access, control, and confidentiality. A blockchain-enabled healthcare infrastructure guarantees that medical health records are integral and interoperable, increases the quality of insurance claim adjudication, and delivers high-quality patient-centered services. Blockchain not only aims to address data protection issues in this regard, but it can also guarantee data privacy, accountability, and shared access [15].

As per the findings of the study by Tariq et al. [34], one of the ways in which blockchain has been making its place in the healthcare system is by ensuring greater security for the healthcare data. It has been asserted that healthcare data is highly vulnerable to privacy, especially, as more and more information is being stored using cloud technologies on a daily basis. As a result, the challenges pertinent to the leakage of sensitive and confidential data are rising. Hence, there is a need to develop healthcare systems that no one can intervene for any purpose not relevant to the purpose for which the data was stored. Moreover, in both existing frameworks and protection mechanisms, centralized architectures are commonly used. Therefore, the successful integration of interoperability between healthcare systems is complex. This implies that it is still a big obstacle for consumers to have full access to private health records. The significant finding of the study by Tariq et al. [34] is that IoT powers the conventional security systems and the mechanisms incorporated by the healthcare institutions, and they cannot address all the security requirements. Thus, in the context of smart cities, blockchain systems can be incorporated to overcome security issues.

The rationale for the incorporation of the blockchain technology for integrating smart city initiatives along with the conventional healthcare practices is presented by the study by Karale and Ranaware [2] that posited that healthcare is one of the potential areas where the application of the technology can be established to ensure greater efficiency. The benefits pointed out in the study go beyond just the security issues. The study further posited that by incorporating this technology, a single electronic health record for all the patients can be created. Such a system would be more trustworthy for both the patients and healthcare professionals. The conventional centralized records are replaced with the decentralized reports that the authorized people, including the patient, can access. The patients are, thus, not required to carry multiple health records at every visit. This study also posited that a database for the professional care providers of the city can be developed. Thus, the hospital staff can be mindful of the available healthcare professionals in the city. Lastly, open pharmaceutical supply chains can be developed where all the operations are carried out by smart contracts [2].

In this context, the study by Vazirani et al. [54] has also put forward blockchain for better interpretability of the information. The study put forward that quick access to an entire collection of medical data will allow clinicians to treat patients without having to wait until prior reports have arrived. The availability of timely and more regular data will allow doctors to draw up specialized care plans based on outcomes and effectiveness of treatment. Traditional health knowledge will also engage a patient further in their own health treatment, and a historic challenge in the area would promote patient compliance. The study further posits that as a result of this, the potential of precision medicine will also be enhanced since a centralized entry point is provided for each patient with all real-time health details. Data obtained from wearable devices and smartphone applications can provide information on the costs and effects of therapies and outcome measurements identified by patients [55]. Along with blockchain technology, fog computing is another technology used to make the healthcare system smarter and more efficient. In the context of smart cities, fog computing is comprised of a range of intelligent technologies, including data storage, data acquisition, and networking. As per Badidi et al. [44] with conventional cloud computing and IoT technology, when an application initiates an operation, the delay period is high. However, in the medical field, reduced latency is important. In this regard, fog computing seems to have good advantages. It reduces service delays compared to the cloud that is characterized by higher latency periods for comprehensive computing and storage [44].

In this context, Kraemer et al. [46] have presented the findings that in healthcare systems, sensor-to-cloud architecture is employed for communication. It is using such a system data from different places using sensors enabling the large-scale data sets. However, in the context of healthcare informatics, the simple sensor-to-cloud architecture sometimes is not suitable. In some healthcare systems, some regulation restricts the management from storing patients' information outside of the healthcare institution. Thus, relying entirely on remote data centers cannot work for contemporary healthcare providers. In this regard, fog computing is one possible way to fill the difference between sensors and analytics in health informatics. This computational versatility opens up new doors for addressing healthcare issues. Efficient patient mobility and improved integration will allow for constant surveillance [46].

In the context of remote monitoring, Gia [55] proposed low-cost remote health monitoring IoT-based system that is powered by fog computing and sensors. The system is developed to collect and store data such as biosignals (i.e., ECG and respiration) and spatial data (i.e., atmospheric temperature and humidity). This data can be distributed wirelessly for real-time and remote control. Also, including fog computing technology in the system would allow the healthcare providers to enhance the efficiency of healthcare services, such as collecting data, categorizing data, push notification, and managing the information channels. Moreover, employing sensor nodes with fog computing, the healthcare providers will develop a low-cost system as the sensor node can run for an extended period of time, up to 155 hours, coupled with low energy consumption [56].  Table 1 illustrates the summary of the findings of the aforementioned selected articles.

## 4. Discussion

This section is dedicated to assessing and analyzing the insights and findings obtained from the systematic review of the relevant secondary literature. The section is divided into three subsections; the first delineates the impact and the potential of the IoT on the healthcare sector; the second delineates the impacts of blockchain on the healthcare sector; the third subsection elucidates the implications of fog computing on the healthcare sector. The whole discussion is intended to carry out in the context of the smart communities.

### 4.1. Impact of IoT on the Healthcare

IoT has been the driving force of smart city initiatives across industries, including healthcare. It has enabled healthcare professionals and organizations to achieve accuracy and reliability in their routine activities [58]. A huge portion of the literature directs the attention toward the fact that the adoption of the IoT is worthy of making its place in the healthcare industry [59, 60]. The use of IoT for the diagnosis, supervision, and treatment of chronic health problems where particular consideration has been paid to stable conditions involving regular monitoring and recording healthcare is confirmed by a substantial portion of such literature [61]. The systematic review, however, revealed that the various inefficiencies pertinent to the technology, are acting as barriers to the more competent management of the healthcare operations and practices. This is why it is asserted that still there is room for greater efficiency and more intelligent operation in the sector. In addition to the lack of safe web interfaces and the absence of transport encryption, there are many IoT information management problems in the healthcare sector [62]. From the systematic review of the relevant literature, IoT has been found to be lacking behind in various areas such as ensuring protection and the privacy of the sensitive and personal data of the patients stored by the hospital, which can be subjected to data breaches, theft, and loss.

### 4.2. Impact of Blockchain on the Healthcare

One of the major concerns in the healthcare sector is found to be the protection and the privacy of the large volumes of the patients' data and healthcare records that are stored by the healthcare institutions [63]. The cases of data breaches, theft, and losses in the healthcare sector have become one typical instance. The data is susceptible as it consists of data pertinent to the identity of the individuals [64]. In this regard, privacy as well as ensuring the integrity of such data has been becoming an important focus. It has been asserted that to ensure the protection and the confidentiality of the data, there is a need to have such sensor contingencies that can guarantee that the records are not being altered, lost, or stolen. In this regard, from the analysis of the relevant literature, it has been found that the incorporation of blockchain technology can effectively address this concern. The transaction blocks created in the blockchain are tied together in a chain and each block is comprised of a combination of its own and the hash of the previous block. Thus, this makes it impossible to steal or alter the data without getting caught. Also, the data can only be accessed by the authorized parties that have the key. By employing blockchain technology in the healthcare system, care providers can create a decentralized but highly protected storage for their healthcare data. The storage can only be accessed by authorized people [65]. Thus, this solves the issue of data breach threats and confidentiality and also eases the accessibility of the data.

Moreover, along with solving the privacy concerns, the incorporation of blockchain technology in the infrastructure of the healthcare institutions guarantees that all data and documents such as medical health records are integral and interoperable. This increases the consistency of insurance claim adjudication and delivers high-quality patient-oriented practices and services. In this respect, blockchain addresses data protection issues and guarantees integrity, accountability, and mutual access to data. The incorporation of blockchain also promotes a better management infrastructure that, by providing a decentralized and transparent data structure, allows the management and access of fragmented patient data [66]. This implies that the capabilities of blockchain technology can be integrated to streamline healthcare practices.

### 4.3. Impact of Fog and Cloud Computing on the Healthcare

The high cost of healthcare services has remained another primary concern of the care providers. Also, the dispersed medical services and data, as well as the rise in the number of people suffering from various medical conditions, lead to a high cost of medical practices. The care providers have been incorporating IoT technology and cloud computing to reduce the cost of operations. Nonetheless, in the context of smart cities, the incorporation of fog computing has been emerging as another relevant and promising technology for incorporating smart city initiatives in healthcare [67]. The systematic review revealed that fog computing is a combination of various smart technologies. In healthcare, data is stored at different places for which cloud-based architecture is employed [68, 69, 71]. Such a system is characterized by multiple issues such as high latency and legal subjections. Thus, remote data centers need to be replaced with smarter technologies. In this regard, it is worth noting that fog computing is comprised of a range of smart devices and computing technologies; thus, this results in the reduction of the time it takes to respond from request to request. Each of the devices in the system acts as processing nodes and, thus, simultaneously manages tasks. This leads to a free cloud pipeline which reduced the latency period. Hence, this technology would guarantee increased efficiency in the practices of healthcare institutes. Moreover, it is asserted that fog computing would allow for affordable access to highly advanced information storage capability [70]. This was well supported by the findings of the systematic review that revealed that fog computing paves the way for low-cost remote health monitoring due to increased efficiency and low energy consumption.

## 5. Conclusions

The paper attempted to conduct a systematic review of the documents pertaining to the impact of the IoT, blockchain, and fog on the healthcare systems and practices in the context of smart cities. Due to the very little availability of relevant data, 10 studies were selected for the review and their findings have been analyzed. It was found from the systematic review that IoT has been the most applied technology among the three by the healthcare sector in smart cities. The smart city has been understood as a geographical area characterized by emerging information and communication technologies facilitating the flow and exchange of information. Thus, with the incorporation of information and communication technologies, the efficiency of the information exchange increases in terms of both cost and speed. In order to support healthcare in the context of smart cities and incorporating smart initiatives, IoT, blockchain technology, and fog computing appear to be quite relevant. The application of these technologies can automate the processes and support healthcare in smart cities. To conceptualize, IoT can be understood as the combination of devices that can interact with each other for sharing and exchanging information. The blockchain has been understood as a distributed database comprising a chain of blocks whereby each block represents a different transaction that acts as a public ledger. Lastly, fog computing is understood as a virtual platform between the computing device and the cloud center.

From the systematic review of the literature, it was found that IoT is the most employed technology by healthcare institutes. IoT has made healthcare operations efficient by enabling efficient and smart diagnosis, supervision, and treatment of medical conditions. However, it was found that despite the abundance of benefits, there is still room for improvement that can be done with the incorporation of other more advanced technologies. The gap exists in streamlining practices, cost efficiency, data privacy, and interoperability of data. In this recognition, blockchain technology and fog computing have been found to be more relevant to the healthcare sector in smart cities. Blockchain technology offers data storage that is highly protected due to chained blocks. As each block is comprised of the hash of the previous block, the stored data cannot be lost, stolen, or altered without being noticed. Also, as the blockchain data can be accessed by the authorized parties that have the key, this enables the care providers to create a decentralized data storage that the authorized parties can only access. Thus, this solves the issue of accessibility of the data by the patients and the issue of data breach and theft.

Moreover, such storage enables the care providers to ensure the interoperability of data. Similarly, fog computing is also found to be driving greater efficiency in healthcare. Fog computing has enabled the care providers to incorporate low-cost remote monitoring coupled with the speed of operations and reduced latency, which could not have been achieved with only IoT technology and conventional cloud computing.

## Figures and Tables

**Figure 1:** Blocks in blockchain (Source: Yaga et al. [26]).

**Figure 2:** Block structure (Source: Zheng et al. [25]).

**Figure 3:** IoT architecture (Source: Patel and Patel [31]).

**Figure 4:** Structure of fog computing (Source: Cha et al. [43]).

**Figure 5:** PRISMA process.

**Table 1:** Summary of the findings of the selected articles.

Year	Title of the article	Author (s)	Findings and results
2019	Smart city and smart-health framework, challenges and opportunities	Al-Azzam and Alazzam [17]	ICT has led to the emergence of smart communities in the context of the healthcare sector. In this regard, with the incorporation of technology, continuous surveillance of patients is possible. This helps identify the critical situation in which immediate intervention is required, such as attending to patients and making changes to the healthcare regulations.

2017	Internet of things for smart healthcare: Technologies, challenges, and opportunities	Baker et al. [30]	The introduction of IoT has enabled healthcare practitioners to incorporate big data and self-learning systems in healthcare. This led to smarter management of the healthcare practices as self-learning systems can learn and intervene in various crucial situations. Thus, with this, the practitioners can determine anomalies timely and take preventive actions. Moreover, due to big data, the care providers can use patients' related data for offering to personalize care to them. However, such systems can be threatening to the sensitive and personal data stored by the hospital and can be subjected to a data breach.

2019	Smart healthcare challenges and potential solutions using the Internet of things (IoT) and big data analytics	Zeadally et al. [57]	IoT allows remote healthcare monitoring to monitor the less or noncritical patients and prescribe treatment remotely. Hence, people living in rural areas can be benefited from this, thus, improving healthcare access and providing better control to the people over their healthcare.

2020	Blockchain as a driver for smart city development: Application fields and a comprehensive research agenda	Treiblmaier et al. [15]	Healthcare institutions have to deal with vast amounts of data of the patients shared with various institutions such as insurance companies. Thus, they are obliged to ensure confidentiality and protect such data, which is the major concern. Ensuring privacy and security for such large amounts of data is not possible with only IoT. In this regard, blockchain technology is increasingly being incorporated to ensure the interoperability of healthcare data.

2020	Blockchain and smart healthcare security: A survey	Tariq et al. [34]	Blockchain ensures high and unbreakable security for healthcare data, which can be subjected to theft and breach. The decentralized storage prevents the intervention by any unauthorized party, and thus, the data cannot be stolen or altered by such parties. Also, in the conventional centralized data systems, there is an issue pertinent to access that can be solved by the incorporation of blockchain technology.

2019	Applications of blockchain technology in smart city development: A research	Karale and Ranaware [2]	The benefits of the blockchain in the healthcare sector transcend beyond just security and privacy concerns. The technology allows for the development of a single healthcare data storage that can be easily accessed by the care providers and the patients. Hence, the patients are not required to carry multiple health records at every visit. The data can also be comprised of all the healthcare professionals in the city and other data pertinent to healthcare.

2019	Implementing blockchains for efficient health care: A systematic review	Vazirani et al. [54]	Blockchain would allow the care providers to get real-time health details, enhancing the effectiveness of precision medicine. Moreover, data from wearable devices and smartphones can be integrated to obtain real-time data. Hence, large amounts of real-time data can be obtained from patients without waiting until prior reports have arrived.

2020	Fog computing for smart cities' big data management and analytics: A review	Badidi, Mahrez and Sabir [44]	Cloud computing and IoT technology are characterized by high latency time, which can be solved by incorporating fog computing. The technology ensures greater efficiency with reduced latency times.

2017	Fog computing in healthcare—a review and discussion	Kraemer, et al. [46]	Conventionally, sensor-to-cloud architecture is used in the healthcare sector for information exchange and accessing information from different locations. This type of infrastructure is restricted by the sector regulation that restricts the management from storing patients' data outside of the healthcare institution. In this regard, fog computing seems promising with a streamlined information exchange process.

2017	Low-cost fog-assisted health-care IoT system with energy-efficient sensor nodes	Gia [55]	Fog computing allows for low-cost remote health monitoring with high speed and efficiency and low energy consumption. Hence, the efficiency of healthcare operations and practices has increased including collecting data, categorizing data and push notification, and managing the information channels.

## Data Availability

The data supporting the findings of this work are available within the article.

## Appendix

### AMSTAR Results

**Table:**

Blockchain, IoT and fog computing for healthcare service in smart cities	
Moderate quality review	
1. Did the research questions and inclusion criteria for the review include the components of PICO?	Partially yes
2. Did the report of the review contain an explicit statement that the review methods were established prior to the conduct of the review and did the report justify any significant deviations from the protocol?	Yes
3. Did the review authors explain their selection of the study designs for inclusion in the review?	Yes
4. Did the review authors use a comprehensive literature search strategy?	Yes
5. Did the review authors perform study selection in duplicate?	No
6. Did the review authors perform data extraction in duplicate?	No
7. Did the review authors provide a list of excluded studies and justify the exclusions?	Yes
8. Did the review authors describe the included studies in adequate detail?	Yes
9. Did the review authors use a satisfactory technique for assessing the risk of bias (RoB) in individual studies that were included in the review?	Partially yes
10. Did the review authors report on the sources of funding for the studies included in the review?	Yes
11. Did the review authors report any potential sources of conflict of interest, including any funding they received for conducting the review?	Yes
	No conflict reported
